# Functional Analysis of Serum Long Noncoding RNAs in Patients with Atrial Fibrillation

**DOI:** 10.1155/2022/2799123

**Published:** 2022-05-16

**Authors:** Qi Zhang, Jun Wang, Ying Wang, Ji-Meng Yang, Hai-Cui Dong, Di Xu

**Affiliations:** ^1^Department of Cardiology, The Affiliated Jiangning Hospital of Nanjing Medical University, Nanjing, China; ^2^Department of Cardiology, The First Affiliated Hospital of Nanjing Medical University, Nanjing, China

## Abstract

**Objectives:**

Long noncoding RNAs (lncRNAs) are closely related to diverse diseases. However, its role in atrial fibrillation (AF) pathogenesis needs further exploration.

**Design:**

We performed microarray analysis on the serum samples from 70 healthy volunteers and 70 AF patients. This study was aimed at detecting the levels of serum lncRNAs and mRNAs and bioinformatically analyze them to establish potential marker(s) for AF diagnosis. Receiver operating curve (ROC) and area under the curve (AUC) were employed to address the AF diagnostic power of lncRNAs.

**Results:**

In the AF serum samples, 753 lncRNAs and 802 mRNAs (*p* ≤ 0.05; fold change ≥ 2) were upregulated, and 315 lncRNAs and 153 mRNAs were downregulated, as opposed to healthy serum samples. Using bioinformatic analysis, we analyzed the top 4 differentially expressed (DE) lncRNAs, namely, *NR-001587*, *NR-015407*, *NR-038455*, and *NR-038894*, and found that the PI3K-AKT cell proliferation signaling pathway was most affected. This was in accordance with our functional analysis of DE mRNAs and adjacent lncRNAs. Notably, the elevated serum *NR-001587* levels were strongly associated with AF incidence.

**Conclusions:**

Our work highlights the role of lncRNAs in AF pathogenesis and provides a novel serum biomarker for AF diagnosis.

## 1. Introduction

Atrial fibrillation (AF) is manifested by rapid irregular atrial events that can end in death [1]. Cardiac diseases and other external triggers can markedly elevate AF risk [2, 3]. Interestingly, AF development can also be attributed to genetic variation. Emerging evidences reveal that AF familial patients exhibit a higher incidence and younger age onset, compared to nonfamilial AF patients [4, 5]. Unfortunately, the underlying mechanism of AF onset is unclear. As such, AF diagnosis and treatment remain suboptimal.

Long noncoding RNAs (lncRNAs), a vital member of the noncoding RNA family, lack coding potential and have low evolutionary conservation, which is defined as transcripts longer than 200 nucleotides [6]. lncRNAs modulate gene transcription via interaction with enhancer or transcriptional factors and regulate miRNA functions via pre-mRNA splicing or sequestering miRNA activity. Previous studies reported that lncRNAs play critical roles in various cardiovascular diseases, such as cardiac hypertrophy and coronary artery disease [7, 8]. Moreover, several lncRNAs in atrial and epicardial adipose tissues are known to associate with AF development [9, 10]. However, there are very limited researches on the expression profiles of lncRNAs in serum of AF patients.

In this study, we performed microarray analysis on serum samples from AF patients and healthy volunteers. Based on our analysis, several lncRNAs were strongly related to AF pathogenesis via well-known AF-related pathways. This information provides us with novel insights into the diagnosis and therapeutic aspects of AF management.

## 2. Methods and Materials

### 2.1. Patients and Samples

Study participants were selected from the Department of Cardiology at the Affiliated Jiangning Hospital of Nanjing Medical University between January 2018 and December 2019. We received informed consent from all participants before the initiation of this study. Serum samples were obtained from patients with chronic nonvalvular AF (*n* = 70) and normal sinus rhythm (SR) (*n* = 70). Chronic AF was described as a persisting episode that lasts >7 days. The selected AF patients had an average age of 55 ± 5 years and did not suffer from hypertension, diabetes, hyperthyroidism, or other heart diseases. Upon serum extraction, samples were transported in liquid nitrogen and were maintained at -80°C for subsequent analyses.

### 2.2. Microarray Expression Profiling of lncRNAs and mRNAs

Agilent Human lncRNA Microarray v 4.0 was used to examine human lncRNAs and mRNAs from AF patients and healthy volunteers at the KangChen Bio-tech Laboratory in Shanghai, China, using operational guidelines. In short, total RNA was converted to cDNA and then to cRNA harboring cyanine-3-CTP. Subsequently, the color-coded cDNAs underwent hybridization with a human lncRNA array consisting of 78,243 lncRNAs and 30,215 mRNAs. Finally, the array was rinsed and scanned by the Agilent Scanner G2505C (Agilent Technologies, USA). The Feature Extraction Software (version 10.7.1.1, Agilent Technologies) was used to analyze array images and extract raw data, which underwent additional analysis in GeneSpring (version 12.5, Agilent Technologies). We normalized the raw data and adjusted the cut-off point to >2.0 and *p* value to <0.05 to detect high- and low-expression genes. Next, we used hierarchical clustering to identify relevant lncRNA and mRNA expression.

### 2.3. Gene Ontology (GO) and Kyoto Encyclopedia of Genes and Genomes (KEGG) Pathway Analyses

GO analysis (http://geneontology.org/) identifies significant gene products involved in three main categories, namely, biological process (BP), cellular components (CC), and molecular function (MF). KEGG (genome.jp/kegg/) predicts molecular binding and signaling pathways related to differentially expressed (DE) genes. The enrichment score (-log10 (*p* value)) signifies the importance of GO term or network enrichment among genes.

### 2.4. Annotation for lncRNA/miRNA/mRNA Interactions

Here, lncRNA, miRNA, and mRNA interactions were estimated using the Arraystar's home-made miRNA target prediction software, based on miRanda (http://microrna.org/microrna/home.do) and TargetScan (http://targetscan.org/vert_71/) [11]. We adjusted the match score to >150 and the minimum free energy to <-25 to enhance prediction reliability. In subsequent analysis, we only chose miRNAs and mRNAs that were identified in both predicted results.

### 2.5. Cis-Acting lncRNA Prediction

We selected two parameters for the prediction of cis-acting lncRNAs: [1] the lncRNA and mRNAs must be adjacent (i.e., within 1,000,000 base pairs), and [2] the lncRNA and mRNAs must present strongly associated profiles (i.e., Pearson correlation coefficient > 0.6 or <−0.6).

### 2.6. Total RNA Extraction and Reverse Transcription-Quantitative Polymerase Chain Reaction (qRT-PCR)

We isolated total RNA from 200 ml of serum and plasma using the miRNeasy kit (Qiagen, Valencia, CA), as reported before [12]. Next, we performed qRT-PCR using the ABI QuantStudio™ 6 Flex Real-time PCR systems, following operational guidelines. The comparative cycle threshold (Ct) formula was utilized for relative gene expression determination. Primers employed in this study are presented in Table 1.

### 2.7. Statistical Analysis

All data analyses were conducted in SPSS 16.0 and are expressed as means ± SD or numbers. Data analyses were done using paired *t* test or chi-squared test. *p* value < 0.05 was set as the significance threshold. lncRNAs with fold change ≥ 2 and *p* value ≤ 0.05 were deemed to be significant. The AF diagnostic value of serum lncRNAs was determined with receiver operating curve (ROC) analysis, using optimal threshold values. The *y*-axis illustrates sensitivity, whereas the *x*-axis illustrates specificity.

## 3. Results

### 3.1. lncRNA and mRNA Expression Profiles in AF Patients and Healthy Individuals

We collected serum samples from AF patients and healthy individuals, and 3 random samples from each group were selected for microarray analysis of lncRNA and mRNAs. 12,956 lncRNAs and 21,975 mRNAs were identified in the serum of AF patients. In addition, 17,342 lncRNAs and 32,524 mRNAs were detected in the serum of healthy individuals (Figures 1(a) and 1(b)). Upon further analysis, 1,068 lncRNAs were identified as DE (*p* ≤ 0.05; fold change ≥ 2). Among them, 753 were upregulated and 315 were downregulated. Likewise, 955 mRNAs were DE, among which 802 were elevated and 153 were reduced in the AF patients compared with healthy controls (Figures 1(c) and 1(d)).

Based on the positioning of lncRNAs in a genome, lncRNAs can be placed under six categories: bidirectional, exon sense-overlapping, intergenic, intro sense-overlapping, intronic antisense, and natural antisense. The aforementioned DE lncRNAs primarily belonged to either exon sense-overlapping (39%) or intergenic (30%), which is consistent with prior reports (Figure 1(e)) [6]. Furthermore, we demonstrated that the distribution of upregulated lncRNAs was in accordance with downregulated lncRNAs (data not shown).

To validate the conclusions of our microarray analysis, we selected 3 (*NR-038435*, *NR-001587*, and *NR-015407*) most upregulated and 3 (*NR-131216*, *NR-038455*, and *NR-038894*) most downregulated lncRNAs which were identified in microarray analysis. The expression profiles of these lncRNAs in 17 randomly picked samples were examined using qRT-PCR assay. Based on our results, expressions of all 6 lncRNAs were consistent with our microarray results, suggesting optimal quality of our microarray analysis. As such, the following bioinformatic analysis can be considered highly credible (Figure 1(f)).

### 3.2. DE mRNA Pathway Analysis

We employed both GO and KEGG analyses to explore the association between DE mRNAs and AF. Using GO analysis, we showed that the elevated mRNAs were involved in cell division (GO:0051301), mitotic nuclear division (GO:0007067), and cell proliferation (GO:0008283) (Figure 2(a)). Meanwhile, downregulated mRNAs were related to the extracellular matrix organization (GO:0030198), angiogenesis (GO:0001525), and insulin receptor signaling pathway (GO:0008286) (Figure 2(b)). We also identified that the most enriched BPs of DE mRNAs were similar to the upregulated mRNAs, suggesting that the upregulated mRNAs are primarily responsible for AF pathogenesis (Figure 2(c)).

Using KEGG analysis, we revealed that the upregulated mRNAs were enriched in the metabolic pathway (hsa01100), cell cycle (hsa04110), and carbon metabolism (hsa01200) (Figure 2(d)). In contrast, the downregulated mRNAs were enriched in purine metabolism (hsa00230), transcriptional misregulation in cancer (hsa05202), and fatty acid metabolism (hsa01212) (Figure 2(e)). Moreover, all DE mRNAs were involved in the metabolic pathway (hsa01100), cell cycle (hsa04110), and biosynthesis of antibiotics (hsa01130) (Figure 2(f)). The above results suggest that the pathways most related to AF are metabolic and cell cycle pathways.

### 3.3. lncRNAs Regulate AF via Sponging miRNAs

It is well-known that lncRNAs modulate BP via sponging miRNAs. To identify relevant downstream miRNAs and target mRNAs, we selected 2 most upregulated lncRNAs, namely, *NR-001587* and *NR-015407*, and 2 most downregulated lncRNAs, namely, *NR-038455* and *NR-038894*, for further analysis (Figure 3). Using GO analysis, we revealed that the most enriched BPs were the positive modulation of GTPase activity (GO:0043547), viral defense pathway (GO:0051607), and negative modulation of viral genome replication (GO:0045071). Among the most enriched CCs were cell-cell junction (GO:0005911) and excitatory synapse (GO:0060076). Lastly, among the most enriched MFs were GTPase activator activity (GO:0005096), syntaxin-1 interaction (GO:0017075), and ribonuclease activity (GO:0004540) (Figures 4(a)–4(c)). Using KEGG analysis, we showed that lncRNAs primarily regulated AF via the PI3K-Akt network (hsa04151), proteoglycans in cancer (hsa05205), and focal adhesion (hsa04510) (Figure 4(d)). Taken together, the above results suggest that the GTPase-PI3K-AKT axis is crucial in the lncRNA-mediated regulation of miRNA activity and, ultimately, AF.

### 3.4. lncRNAs Modulate AF via Adjacent mRNAs

Another well-known notion is that lncRNAs modulate adjacent mRNA expression in a cis-acting manner [13]. To establish biological lncRNA and mRNA pairs, we first identified DE lncRNAs and mRNAs and then screened for lncRNAs containing adjacent mRNAs (within one million base pairs). Based on our analysis, we discovered 140 lncRNA-mRNA pairs. Among them, 58.5% (82 in 140) pairs exhibited positive correlations. Exon sense-overlapping (50%) and intergenic (37.5%) accounted for the majority lncRNA-mRNA pairs, which is consistent with the distribution of overall DE lncRNAs (Figure 5(a)).

We next conducted both GO and KEGG analyses on the identified lncRNA-mRNA pairs. GO analysis revealed that the most enriched BPs were cellular protein metabolic process (GO:0044267), cell division (GO:0051301), and positive modulation of NF-kappa B transcription factor activity (GO:0051092). The most enriched CCs were extracellular region (GO:0005576) and cell surface (GO:0009986). Lastly, the most enriched MFs were protein heterodimerization activity (GO:0046982), cytokine activity (GO:0005125), and histone binding (GO:0042393) (Figures 5(b)–5(d)). Using KEGG analysis, we revealed that lncRNAs modulate AF via the PI3K-Akt network (hsa04151), alcoholism (hsa05034), and systemic lupus erythematosus (hsa05322) (Figure 5(e)). These results further validate that the GTPase-PI3K-AKT-cell proliferation axis is strongly associated with AF.

### 3.5. The AF Diagnostic Power of Serum lncRNAs

The above results demonstrated that serum lncRNAs are strongly related to AF incidence. To further address the AF diagnostic power of lncRNA, we collected an additional 50 blood samples from AF patients and healthy individuals. qRT-PCR was employed to detect 4 most DE lncRNAs, namely, *NR-001587*, *NR-015407*, *NR-038455*, and *NR-038894*. Based on our data, all 4 lncRNAs were associated with AF (Figure 6(a)). Then, we performed ROC analysis to determine the potential diagnostic power of these 4 lncRNAs. Our data revealed that the AUC of NR-001587 was 0.815 (95% CI 0.722-0.908), with 84% sensitivity and 86% specificity (cut-off value was 1.582). The AUC of NR-015407 was 0.630 (95% CI 0.519-0.741) with 86% sensitivity and 42% specificity (cut-off value was 1.082). The AUC of NR-038455 was 0.673 (95% CI 0.566-0.780), with 72% sensitivity and 64% specificity (cut-off value was 0.665). Lastly, the AUC of NR-038894 was 0.699 (95% CI 0.594-0.804), with 54% sensitivity and 84% specificity (cut-off value was 0.522) (Figure 6(b)). The above results suggest that serum NR-001587 is an excellent biomarker candidate for AF diagnosis.

## 4. Discussion

AF is a highly prevalent form of cardiac arrhythmia that exerts a massive financial burden on patients. Clinically, an AF patient is treated, according to the CHADS score [14]. Till now, no serum biomarkers have been used to diagnose AF in clinic. This is mostly due to the limited knowledge regarding the molecular mechanism underlying AF pathogenesis. Unfortunately, the lack of knowledge affects not only diagnosis but also treatment of AF. Recently, several studies reported a critical role of lncRNAs in modulating diverse cellular processes, including AF [7, 8, 10, 15]. However, available research on serum lncRNAs and AF is scarce. In our study, we employed bioinformatics to analyze serum lncRNAs from AF patients to identify potential key lncRNAs and underlying mechanisms related to AF development. These lncRNAs may serve as biomarkers for AF status and may aid in the design of personalized treatment plans. Zeng and Jin reported that serum lncRNA ANRIL (antisense noncoding RNA in the INK4 locus) is closely related to AF, with ischemic stroke or recurrence-free survival, indicating that lncRNAs can be effective diagnostic indicators for AF [16].

Here, we analyzed the serum microarray data from AF patients and healthy adults. Consequently, we identified 802 upregulated mRNAs and 153 downregulated mRNAs in AF serum versus healthy controls. Our subsequent functional analysis revealed that cell proliferation is intensively associated with AF pathogenesis. It is well-known that the heart structural and electrophysiological remodeling promotes the onset of AF. Interestingly, AF can also promote heart remodeling of its own, particularly via fibroblast proliferation. Lu et al. reported that lncRNA GAS5 inhibits fibroblast proliferation in AF patients, which, in turn, restores heart function in AF patients [17]. Given these results, suppressing cell proliferation may be a novel therapeutical approach to managing AF.

To elucidate the mechanism whereby DE lncRNAs regulate AF, we employed two methods of screening downstream genes, based on two well-known mechanisms. One involves the possibility that lncRNAs sponge miRNAs to regulate BP, and another involves the lncRNA-mediated regulation of adjacent mRNA expression in a cis-acting manner [13]. Based on our functional analysis of predicted genes, the GTPase-PI3K-AKT axis is strongly correlated with AF pathogenesis. Multiple studies have confirmed that the PI3K-AKT network is related to AF [18–20]. Together with the fact that fibroblast proliferation is associated with the PI3K-AKT network, we hypothesized that the PI3K-AKT-fibroblast proliferation axis might be critical for AF pathogenesis. However, the regulatory mechanism by which DE lncRNA regulates the PI3K-AKT pathway in the AF pathogenesis needs to be elucidated in future studies.

## 5. Conclusion

In summary, our work used microarray analysis to identify serum lncRNAs that are specific to AF diagnosis. Based on our results, the PI3K-AKT-fibroblast proliferation axis was found to be strongly associated with AF pathogenesis. In addition, we demonstrated that NR-001587 can serve as a serum biomarker for AF, owing to its high sensitivity (84%) and specificity (86%). Our work provides a basis for future investigation on the molecular mechanism of the lncRNA-mediated modulation of AF and highlights the potential of serum lncRNA to serve as biomarkers for AF diagnosis.

## Figures and Tables

**Figure 1:** The expression profiles of lncRNAs and mRNAs. (a, b) A heat map showing the expression profiles of differentially expressed (DE) lncRNAs (a) and DE mRNAs (b) in the serum of individuals with A: atrial fibrillation (AF) or without C: control. (c, d) A volcano diagram showing levels of serum lncRNAs (c) and mRNAs (d) in AF and non-AF patients. The green and red bolts represent downregulated and upregulated genes (*p* ≤ 0.05; fold change ≥ 2), respectively. (e) A pie chart representing DE lncRNA distribution, based on their position on the genome. (f) The qRT-PCR-identified expression of 6 lncRNAs, namely, *NR-038435*, *NR-001587*, *NR-015407*, *NR-038455*, *NR-038894*, and *NR-131216* in the serum of AF patients and healthy volunteers. Data are presented as mean ± standard error, *n* = 17, ^∗^*p* < 0.05.

**Figure 2:** Functional analysis of DE mRNAs. (a–c) BP (biological process) enrichment GO analysis illustrating upregulated (a), downregulated (b), and DE mRNAs (c). (d–f) KEGG analysis of upregulated (d), downregulated (e), and DE mRNAs (f).

**Figure 3:** Bioinformatic analysis identifying target miRNAs sequestered by the top 4 lncRNAs from microarray analysis. Yellow dots refer to lncRNAs, red dots refer to miRNAs, and blue dots refer to mRNAs.

**Figure 4:** The functional ceRNA analysis of the top 4 DE lncRNAs. (a–c) BP (biological process) (a), CC (cellular component) (b), and MF (molecular function) (c) of GO analysis of the top 4 DE lncRNAs, namely, *NR-001587*, *NR-015407*, *NR-038455*, and *NR-038894*. (d) KEGG analysis of the top 4 DE lncRNAs.

**Figure 5:** Functional analysis of the predicted lncRNA-mRNA pairs. (a) LncRNA-mRNA pair distributions. (b–d) BP (b), CC (c), and MF (d) of GO analysis examining different lncRNA-mRNA pairs. (e) KEGG analysis of the lncRNA–mRNA pairs.

**Figure 6:** The AF diagnostic power of serum lncRNAs. (a) qRT-PCR analysis of *NR-001587*, *NR-015407*, *NR-038455*, and *NR-038894* in serum of AF patients and healthy counterparts. (b) ROC analysis of serum *NR-001587*, *NR-015407*, *NR-038455*, and *NR-038894* in the diagnosis of AF.

**Table 1:** The primer sequences used in this study to detect differentially expressed lncRNAs.

Names	Primers	Products (bp)
*β*-Actin (H)	F: 5′ GTGGCCGAGGACTTTGATTG3′ R: 5′ CCTGTAACAACGCATCTCATATT3′	73
NR_131216	F: 5′ TGACCATCAGTAAGAGACACGG 3′ R: 5′ TATCCTAGCCTTGGCGAGAG 3′	122
NR_038435	F: 5′ GAAAGTAAATGTCCTTGGCTG 3′ R: 5′ AAGGAAGTGCTATTTCACATCC 3′	152
NR_015407	F: 5′ GTCTAAGGTGGAGATTACCAGG 3′ R: 5′ CCACAGACATCATTACATACGG 3′	59
NR_001587	F: 5′ ACTTTGTGCTGACTCGATCG 3′ R: 5′ AGGTACTTGGAAGGTTATTGG 3′	54
NR_038455	F: 5′ GCAATTCAGCACTTGTCATGC 3′ R: 5′ CAGATATGGTCCTTGCCAGTCT 3′	128
NR_038894	F: 5′ CCTCGTACAGCACGCATTCA 3′ R: 5′ TAGCCGCCAAGTTTCTGAGA 3′	136

## Data Availability

All data was included in our manuscript.
